The article "Oncoproteins of High-Risk HPV and EBV Cooperate to Enhance Cell Motility and Invasion of Human Breast Cancer Cells via Erk1/Erk2 and β-Catenin Signaling Pathways" was retracted in 2021. Reason: concerns about the images.

# Oncoproteins of High-Risk HPV and EBV Cooperate to Enhance Cell Motility and Invasion of Human Breast Cancer Cells *via* Erk1/Erk2 and β-Catenin Signaling Pathways

**DOI:** 10.3389/fonc.2021.630408

**Published:** 2021-03-12

**Authors:** Ishita Gupta, Ayesha Jabeen, Semir Vranic, Ala-Eddin Al Moustafa, Hamda Al-Thawadi

**Affiliations:** ^1^College of Medicine, Qatar University Health, Qatar University, Doha, Qatar; ^2^Biomedical and Pharmaceutical Research Unit, Qatar University Health, Qatar University, Doha, Qatar; ^3^Biomedical Research Centre, Qatar University, Doha, Qatar

**Keywords:** breast cancer, gene deregulation, HPV, EBV, *in-vitro*, oncoproteins

## Abstract

Breast cancer is a leading cause of death in women around the world. Most breast cancer-related deaths are a result of complications from the metastatic spread. Several recent studies reported that high-risk human papillomaviruses (HPVs) and Epstein–Barr virus (EBV) are co-presented in different types of human carcinomas including breast; however, the cooperative effects between high-risk HPVs and EBV oncoproteins in human breast cancer have not been investigated yet. Thus, we herein explored the cooperation outcome between E6/E7 and latent membrane protein 1 (LMP1) oncoproteins of high-risk HPV type 16 and EBV, respectively, in two human breast cancer cell lines, MCF7 and MDA-MB-231. Our data revealed that the cooperation of E6/E7 and LMP1 oncoproteins stimulates cell proliferation and deregulates cell cycle progression of human breast cancer and normal mammary cells; in parallel, we noted that E6/E7/LMP1 incite colony formation of both breast cancer cell lines but not normal cells. More significantly, our results point out that the co-expression of E6/E7 and LMP1 oncoproteins enhances cell motility and invasion of MCF7 and MDA-MB-231 cell lines; this is accompanied by deregulation of epithelial–mesenchymal transition biomarkers including E-cadherin, β-catenin, fascin, and vimentin. The molecular pathway analysis of HPV and EBV oncoproteins cooperation shows that it can enhance the phosphorylation of extracellular signal-regulated kinases (Erk1/Erk2) in addition to β-catenin, which could be behind the effect of this cooperation in our cell models. The study clearly suggests that high-risk HPV and EBV coinfection can play an important role in breast cancer progression *via* Erk1/Erk2 and β-catenin signaling pathways.

## Introduction

Breast cancer, the most commonly diagnosed cancer in women, represents ~25% of all cancer cases (1). While breast cancer is the leading cause of mortality in developing countries (~14%), in developed countries, it is the second cause of cancer-related mortality (~15%) (1). Most breast cancer-related deaths result from complications due to metastasis to vital organs including the brain, bone, liver, and lung (2, 3). Breast cancer is a complex and heterogeneous disease at the molecular level, with different gene expression patterns leading to differences in clinical behaviors and outcomes (4). On the one hand, based on gene expression profiling of human breast tumors, they are classified into four subtypes (luminal A, luminal B, human epidermal growth factor receptor-2 (HER2)-positive, and triple-negative) (5). On the other hand, it has been indicated that gene alteration, lifestyle, and environmental factors play a vital role in breast cancer etiology (6, 7). Additionally, it has been recently pointed out that oncoviruses, such as high-risk human papillomaviruses (HPVs) and Epstein–Barr virus (EBV), can be involved in the onset and progression of breast cancer (8–15).

The article "Oncoproteins of High-Risk HPV and EBV Cooperate to Enhance Cell Motility and Invasion of Human Breast Cancer Cells via Erk1/Erk2 and β-Catenin Signaling Pathways" was retracted in 2021. Reason: concerns about the images.

Globally, it has been shown that high-risk HPVs are present in 2–86% of human breast cancer cases (10, 11, 13, 16–18), while EBV is present in 30–50% of the cases (11, 19–22). However, a few studies have failed to detect the presence of HPV or EBV in breast cancer (23–26). The distribution of HPV in breast cancer varies geographically; different countries including Mexico, China, United Kingdom, Iran, India, Syria, and Qatar reported a prevalence of 40–65% (10, 27–32), while others, such as Japan and Jordan, reported a lower prevalence of around 21% (33, 34). Similarly, a varying frequency of EBV infection has been reported; in Jordan, Pakistan, Portugal, and Eritrea, EBV was present in 24–28% (34), while a higher frequency was reported in Qatar (49%), Syria (52%), and Sudan (53%), respectively (12, 35, 36). Co-presence of HPV and EBV has been reported in breast cancer; coinfection in such cases is significantly higher in cancer when compared to normal breast tissues (11). However, a study in Australia showed co-presence of HPV and EBV in ~76% of breast cancers (11); in Qatar and Syria, coinfection was reported in 47 and 32% of the cases, respectively (14, 32). In Pakistan, a low frequency of 9% was revealed (37). On the other hand, a study in Jordan identified multiple viral infections in 6% of breast cancer cases (34). Moreover, an investigation by Glenn et al. (11) demonstrated the co-presence of HPV and EBV in breast cancer correlated with diagnosis at a younger age and a more aggressive grade of breast cancer.

Nevertheless, it has been established by an earlier study that E6/E7 oncoproteins of high-risk HPV type 16, the most frequent HPV type worldwide, can convert non-invasive and non-metastatic breast cancer cells into invasive and metastatic ones (38). On the other hand, latent membrane protein 1 (LMP1) is one of the major oncoproteins of EBV involved in inducing cellular proliferation and motility as well as restraining apoptosis, thus indicating the role of EBV in carcinogenesis (39, 40). Several recent investigations reported that high-risk HPV and EBV can be co-present in different types of human carcinomas, including cervical, head, and neck, colorectal in addition to the breast (12, 14, 32, 36, 41–46). Moreover, it has been reported that the co-presence of high-risk HPVs and EBV is associated with the tumor grade and stage in addition to positive lymph nodes in breast cancer and other types of human cancers (14, 32, 36, 44–46). However, the outcome of oncoproteins cooperation of high-risk HPVs and EBV in human cancer cells, including breast, has not been explored yet. Therefore, we herein investigated for the first time the cooperative effect of E6/E7 oncoproteins of HPV type 16 and LMP1 of EBV in two human breast cancer cell lines, MCF7 and MDA-MB-231, luminal A and triple negative breast cancer (TNBC), respectively.

The article "Oncoproteins of High-Risk HPV and EBV Cooperate to Enhance Cell Motility and Invasion of Human Breast Cancer Cells via Erk1/Erk2 and β-Catenin Signaling Pathways" was retracted in 2021. Reason: concerns about the images.

Our data point out that these oncoproteins can cooperate to enhance cell proliferation and invasion of both cell lines in comparison with their matched controls. Moreover, our study revealed that this cooperation occurs *via* extracellular signal-regulated kinases (Erk1/Erk2) and β-catenin signaling pathways.

## Materials and Methods

### Cell Culture

Two different breast cancer cell lines (MCF7 and MDA-MB-231) derived from females were purchased from American Type Culture Collection (ATCC, Manassas VA, USA). Cell lines were grown and expanded in the Dulbecco's modified Eagle's medium (DMEM) (Gibco^®^, Life Technologies, Burlington, ON, Canada) supplemented with 10% fetal bovine serum (FBS; Invitrogen, Life Technologies, Burlington, ON, Canada), and 1% penicillin–streptomycin (Pen-Strep) antibiotic (Invitrogen, Life Technologies). We used human normal mammary epithelial (HNME) cells as control. HNME cells were maintained in keratinocyte serum-free medium (KSFM) (1×) (Gibco^®^, Life Technologies) supplemented with 1% Pen-Strep antibiotic (Invitrogen, Life Technologies). Cells were maintained at 37°C and in 5% CO_2_ atmosphere.

### Transduction of Breast Cancer Cells With E6/E7 and LMP1 of HPV-16 and EBV, Respectively

Subconfluent breast cancer cell lines, MCF7 and MDA-MB-231, as well as the control, HNME were transduced by retro-vectors carrying E6/E7 in addition to LMP1, as previously illustrated by our group (47–49). Briefly, HPV E6/E7 and EBV LMP1 open-reading frames (ORFs) were cloned into the murine-based retroviral vector pLXSN (Takara Bio USA, Inc, Mountain View, CA, USA). The constructs were transfected into a packaging cell line PA317, and recombinant retrovirus was collected in the supernatant. The resulting pLXSN virus was used to infect the early passage breast cancer and HNME cells. Cells were selected with G418 at 300 μg/ml and passaged in culture. Over 95% of E6/E7 and LMP1 cancer cells were healthy after the G418 treatment. The transduced cells were subsequently maintained in the long-term culture with the DMEM. The non-transduced breast cancer cells (MCF7 and MDA-MB-231) and HNME cells were used as control. On the one hand, we termed HNME cells as HNME-Control, HNME-E6/E7, HNME-LMP1, and HNME-E6/E7/LMP1. On the other hand, MCF7 cells were termed as MCF7-Control, MCF7-E6/E7, MCF7-LMP1, and MCF7-E6/E7/LMP1, while MDA-MB-231 cells were termed as MDA-Control, MDA-E6/E7, MDA-LMP1, and MDA-E6/E7/LMP1.

The article "Oncoproteins of High-Risk HPV and EBV Cooperate to Enhance Cell Motility and Invasion of Human Breast Cancer Cells via Erk1/Erk2 and β-Catenin Signaling Pathways" was retracted in 2021. Reason: concerns about the images.

As previously demonstrated by our group, normal control cells and normal cells were transduced with pLXSN vector and treated with G418 (38, 47, 50). We found that after the G418 treatment, ~95% of the E6/E7-immortalized cells were healthy (47). E6/E7 and/or LMP1 transduced cells were trypsinized and passaged two times, when maintained on G418 (47). However, the normal cells died after around 4 days of the G418 treatment; pLXSN-transduced cells attained senescence after almost 10 passages (47).

For the transduction experiments, standard biosecurity and institutional safety procedures were followed, and all procedures were ethically approved by the Institutional Biosafety Committee of Qatar University (QU-IBC-2018/22).

### 3-(4,5-Dimethylthiazol-2-yl)-2,5-Diphenyl Tetrazolium Bromide Cell Proliferation Assay

The cell number was determined empirically after testing the proliferative capacity of MCF7 and MDA-MB-231 cell lines in comparison to the HNME cells in the 3-(4,5-dimethylthiazol-2-yl)-2,5-diphenyl tetrazolium bromide (MTT) assays using an increasing number of cells. On the one hand, 10,000 cells (MCF7 and MDA-MB-231) were plated onto a 96-well plate in DMEM supplemented with 10% FBS and left to adhere for 24 h. On the other hand, HNME cells (10,000 cells) were plated into a 96-well plate in KSFM and left to adhere for 24 h. To measure proliferation in each well, 10 μl of an MTT stock solution (5 mg/ml) was added, and the plates were incubated for 4 h at 37°C. This was followed by decanting the culture media from the plates, dissolving the formazan crystals formed with 75 μl of dimethyl sulfoxide (DMSO) with incubation for 5 min, and then measuring the absorbance at 560 nm using a plate reader.

### Cell Cycle Analysis

MCF7, MDA-MB-231, and HNME cell lines were plated in 100 mm dishes (1 × 10^6^ cells/dish) and were allowed to attach for 24 h. The cells were synchronized by culturing them overnight in media with 10% FBS. Then, the cells were washed two times with phosphate-buffered saline (PBS), and the culturing media was replaced with fresh media enriched with 10% FBS. At 24 h, cells were harvested by trypsinization, washed with PBS, and fixed overnight in 70% ice-cold ethanol, and the DNA was stained with propidium iodide after RNAse treatment according to the standard protocol (49). The cell cycle analysis was performed using flow cytometry (BD Biosciences, San Jose, CA, USA), and cells in G0/G1, S, G2/M, and the sub-G0/G1 (apoptotic) phases were quantified.

The article "Oncoproteins of High-Risk HPV and EBV Cooperate to Enhance Cell Motility and Invasion of Human Breast Cancer Cells via Erk1/Erk2 and β-Catenin Signaling Pathways" was retracted in 2021. Reason: concerns about the images.

### Soft Agar Growth Assay

About 5,000 breast cancer cells (control and transduced) were placed in DMEM containing 0.4% agar and plated over a layer of DMEM containing 0.7% agar. Similarly, 2 × 10^3^ HNME cells (control and transduced) were placed in KSFM containing 0.4% agar and plated over a layer of KSFM containing 0.7% agar. The cultures were examined every 1–2 days for 3 weeks.

### Cell Wounding Assay

Control cells (non-transfected) and transfected breast cancer cell lines were seeded in six-well plates (5 × 10^5^ cells/well) and allowed to adhere for 24 h. The cells were kept in 2% FBS overnight for synchronization. Following PBS wash, a sterile pipette tip was used to scratch a vertical line in the middle in each well. The detached cells were then removed by washing with PBS. After washing with PBS, DMEM was added. Cell lines were photographed after 24 h.

### Invasion Assay

The cell invasion assay was carried out in 24-well Biocoat Matrigel Invasion Chambers (pore size of 8 μm, Corning, NY, USA) as per the protocol of the manufacturer. In brief, the bottom chamber was filled with DMEM supplemented with 10% FBS, and the upper chamber was seeded with 5 × 10^4^ of different cell lines in the media without FBS and then incubated at 37°C. After 24-h incubation, non-invasive cells were scraped with a cotton swab, and cells that migrated to the lower surface of the membrane were fixed with methanol and stained with 0.4% crystal violet. For quantification, cells were counted under the microscope in five predetermined fields as previously described (49). The percentage of cell invasion was calculated with their matched control. Each experiment was carried out in triplicates.

### Preparation of RNA Samples and Reverse Transcription-PCR

Total RNA was isolated using the RNeasy Mini Kit (Qiagen, Valencia, CA, USA) from both control and transfected cells (E6/E7, LMP1, and E6/E7 + LMP1) according to the instructions of the manufacturer. For the reverse transcription (RT)-PCR analysis, 100 ng of total RNA was reverse transcribed using SuperScript™ III One-Step RT-PCR System with Platinum™ *Taq* DNA Polymerase (Thermo Fisher Scientific, Waltham, MA, USA). Samples were incubated in the Proflex Thermal Cycler (Thermo Fisher Scientific, Waltham, MA, USA) for reverse transcription at 60°C for 30 min, initial PCR activation step at 94°C for 2 min followed by 40 PCR cycles. Each cycle consisted of annealing at 94°C for 15 s, at 61°C for 30 s, and at 68°C for 1 min. Final annealing was at 68°C for 5 min. The oligonucleotide primers used in this study have been described previously (45, 51). The RT-PCR products were examined by electrophoresis on 1% agarose gel containing 0.2 μg/ml ethidium bromide.

The article "Oncoproteins of High-Risk HPV and EBV Cooperate to Enhance Cell Motility and Invasion of Human Breast Cancer Cells via Erk1/Erk2 and β-Catenin Signaling Pathways" was retracted in 2021. Reason: concerns about the images.

### Western Blot Analysis

Total cell lysates from the control and transduced breast cancer cell lines were collected using the radioimmunoprecipitation assay (RIPA) buffer (Santa Cruz Biotechnology, Inc., Dallas, TX, USA). The lysate was incubated on ice for 30 min and vortexed briefly every 10 min, and then centrifuged at 17,000 × *g* for 15 min to collect the proteins. The final protein concentration in the supernatant was determined using the BCA Assay Reagent (Pierce Biotechnology, Waltham, MA, USA). Equal amounts (30 μg) of total cell extracts were boiled for 5 min in an equal volume of reducing buffer, resolved on 10% polyacrylamide gels, and electroblotted onto nitrocellulose membranes. The membranes were probed with a number of primary antibodies as follows: anti-mouse E-cadherin (Abcam, Cambridge, UK: abID# ab1416), anti-rabbit β-catenin (CST 9562), anti-rabbit phosphorylated β-catenin (CST 4176), anti-rabbit Fascin (Abcam: abID# ab183891), anti-rabbit Vimentin (Abcam: abID# 92547), anti-rabbit anti-ERK1/ERK2 antibody (Abcam: abID# ab17942), and anti-rabbit phosphorylated ERK1/ERK2 (Abcam: abID# ab201015). Equal loading of the protein samples was assessed by reprobing the membrane with anti-rabbit glyceraldehyde 3-phosphate dehydrogenase (GAPDH) antibody (Abcam: abID# 9485). Immunoreactivity was detected using chemiluminescence as recommended by the manufacturer (Pierce Biotechnology, Waltham, MA, USA).

In order to obtain a relative quantification of gene expressions, images acquired from Western blotting were analyzed using ImageJ software (National Institutes of Health, Bethesda, MD, USA). The intensity of the bands relative to the GAPDH bands was used to calculate a relative expression of proteins in each cell line.

### Statistical Analysis

Results were presented as mean ± SEM of triplicates from three experiments, and the data were analyzed statistically using one-way ANOVA and *post-hoc* test (multiple comparisons using the Dunnett's test) using the GraphPad Prism (Version 8.4.3, San Diego, CA, USA). Differences with *p* < 0.05 were considered significant.

The article "Oncoproteins of High-Risk HPV and EBV Cooperate to Enhance Cell Motility and Invasion of Human Breast Cancer Cells via Erk1/Erk2 and β-Catenin Signaling Pathways" was retracted in 2021. Reason: concerns about the images.

## Results

To assess the role of oncoviruses coinfection (high-risk HPVs and EBV) in human breast cancer, we examined the cooperative effects of E6/E7 of HPV type 16 and LMP1 of EBV on selected parameters in two breast cancer cell lines, MCF7 and MDA-MB-231. HNME cells were used as control. We transduced MCF7, MDA-MB-231, and HNME cells with E6/E7 and LMP1, individually and in combination, using a recombinant retroviral system as described previously (38, 49). In our study, we utilized polyclonal populations of MCF7-E6/E7, MCF-LMP1, MCF7-E6/E7/LMP1, MDA-E6/E7, MDA-LMP1, MDA-E6/E7/LMP1, and HNME (E6/E7, LMP1, and E6/E7/LMP1) cells; we confirmed that these cell lines express E6/E7 and LMP1 in comparison with their wild-type counterparts by RT-PCR (Figure 1).

**Figure 1:** The RT-PCR analysis of E6/E7 and LMP1 expression of HPV and EBV, respectively, in MCF7-Control, MCF7-E6/E7, MCF-LMP1, MCF7-E6/E7/LMP1, MDA-MB-231-Control, MDA-E6/E7, MDA-LMP1 and MDA-E6/E7/LMP1, HNME-Control, HNME-E6/E7, HNME-LMP1, and HNME-E6/E7/LMP1 cells. We note that the cell lines express E6/E7 when transduced with E6/E7 alone and in combination, while LMP1 is present in cell lines transduced with LMP1 alone and in combination. The controls did not express E6/E7 or LMP1.

We initially analyzed the proliferative ability of transduced cell lines in comparison with their wild-type cells using the MTT assay; our data revealed that E6/E7 and LMP1 alone enhance cell proliferation in breast cancer cell lines, whereas the co-presence of E6/E7 and LMP1 induces significant cell proliferation (5-fold, 3.4-fold, and 2-fold) in both breast cancer and normal mammary cells in comparison with cells expressing E6/E7 (2-fold, 1.4-fold, and 1.3-fold) or LPM1 (3-fold, 1.8-fold, and 1-fold) alone in MCF7, MDA-MB-231, and HNME, respectively, and in control cells (Figure 2). Later, we analyzed cell cycle progression of transduced cell lines in comparison with wild-type cells using flow cytometric analysis. Our results showed that E6/E7 and LMP1 oncoproteins together cause a significant increase (1.1-fold, 1.2-fold, and 1.2-fold) in MCF7, MDA-MB-231, and HNME, respectively (*p* = 0.04, *p* = 0.001, and *p* = 0.04) in the percentage of G0 and G1 phase cells in comparison with E6/E7 (1.0-fold, 1.1-fold, and 1.1-fold) or LMP1 (1-fold, 1.1-fold, and 1.2-fold) alone and in control cells, indicating uncontrolled cell growth (Figure 3).

**Figure 2:** Effect of oncoproteins of HPV and EBV (E6/E7 and LMP1, respectively), on cell proliferation of breast cancer cell lines **(A)** MCF7 and **(B)** MDA-MB-231, and **(C)** HNME after 24 h of using the MTT assay. Data are presented in comparison to controls, clearly cell lines that co-express E6/E7 and LMP1 exhibit the highest proliferation rate (*p* < 0.001), whereas LMP1 and E6/E7 induce cell proliferation but to a lesser extent (*p* < 0.001). The data are expressed as a percent of growth ± SEM.

The article "Oncoproteins of High-Risk HPV and EBV Cooperate to Enhance Cell Motility and Invasion of Human Breast Cancer Cells via Erk1/Erk2 and β-Catenin Signaling Pathways" was retracted in 2021. Reason: concerns about the images.

**Figure 3:** Cell cycle analysis of **(A)** MCF7 and **(B)** MDA-MB-231, and **(C)** HNME cells under the effect of E6/E7 and LMP1. Data demonstrate an increase in G0/G1 phase with a simultaneous reduction in S and G2/M phases of both cell lines.

Later, we assessed the colony formation of our cell lines using soft agar assay, which is generally employed to confirm the transformation ability of the cells; we noted a significant increase in the number and size of colonies for both breast cancer cell lines, MCF7 and MDA-MB-231, expressing E6/E7 and LMP1 together (3.8-fold and 7.6-fold) compared to E6/E7 (0.8-fold and 1.2-fold) and LMP1 (1.4-fold and 3.2-fold) alone and their matched controls in MCF7 and MDA-MB-231, respectively as shown in Figures 4A,B. In contrast, HNME cell lines expressing E6/E7 and LMP1 individually and together did not provoke colony formation in soft agar (data not shown). Thus, it is clear that E6/E7 and LMP1 can cooperate in HNME cells to stimulate cell proliferation and deregulate cell cycle progression, but it does not induce cellular transformation of HNME cells.

**Figure 4:** Effect of E6/E7/LMP1 on colony formation, in soft agar, in (**A)** MCF7 and **(B)** MDA-MB-231 cell lines. As shown, E6/E7/LMP1 induces colony formation of MCF7 and MDA-MB-231 cells in comparison with their matched control cell lines; in contrast, E6/E7 and LMP1 are unable to incite HNME cells to form a colony in soft agar (data not shown). Colonies were counted manually and expressed as mean ± SEM.

Based on the above data, we investigated cell motility and invasiveness of transduced breast cancer cell lines and their wild-type cells using wound-healing and invasion assays, respectively. We found that the co-expression of E6/E7 and LMP1 enhances significantly cell motility (0.7-fold and 6.3-fold) and invasive abilities (0.4-fold for each cell line) of both the cell lines, MCF7 and MDA-MB-231, respectively, in comparison with E6/E7 and LMP1 alone and with wild-type cells (Figures 5, 6).

**Figure 5:** Outcome of E6/E7 and LMP1 of HPV16 and EBV, respectively, on cell motility in **(A)** MCF7 and **(B)** MDA-MB-231. We note that cotransduction of E6/E7 and LMP1 enhances cell motility of MCF7 and MDA-MB-231 cell lines in comparison with E6/E7 and LMP1 alone and with their wild-type counterparts.

The article "Oncoproteins of High-Risk HPV and EBV Cooperate to Enhance Cell Motility and Invasion of Human Breast Cancer Cells via Erk1/Erk2 and β-Catenin Signaling Pathways" was retracted in 2021. Reason: concerns about the images.

**Figure 6:** Effect of E6/E7 and LMP1 of HPV16 and EBV, respectively, on cell invasion in both breast cancer cell lines **(A)** MCF7 and **(B)** MDA-MB-231 cells. E6/E7/LMP1 increases cell invasion ability of both cancer cell lines by ~20% in comparison with their matched control cells (*p* < 0.05). The Boyden chambers were used to assess the cell invasion ability of MCF7 and MDA-MB-231 cell lines.

Subsequently, we explored the expression patterns of several important biomarkers of cell invasion and epithelial-mesenchymal transition (EMT), including E-cadherin, β-catenin, vimentin, and fascin genes in our cell line models. On the one hand, our data showed that E6/E7/LMP1 cooperation reduces the expression of E-cadherin and β-catenin in both breast cancer cell lines, MCF7 and MDA-MB-231, in comparison with E6/E7 and LMP1 alone and control cells; on the other hand, vimentin and fascin were significantly upregulated under the effect of E6/E7/LMP1 cooperation as shown in Figure 7.

**Figure 7:** Protein expression and molecular pathways of E6/E7 and LMP1 crosstalk in **(A)** MCF7 and **(B)** MDA-MB-231 cells. E6/E7/LMP1 downregulates E-cadherin and β-catenin and upregulates vimentin and fascin in comparison with their control. Furthermore, E6/E7/LMP1 enhances the phosphorylation of β-catenin, ERK1/2 while slightly increasing the total Erk1/2 expression. β-actin was used as a control in this assay.

*Vis-à-vis* the underlying molecular mechanisms of E6/E7/LMP1 cooperation, we assumed that β-catenin and Erk1/Erk2 signaling pathways could be involved; this was based on our recently published work on HPV and EBV interactions in human cancer and EMT (42, 46, 52, 53). Our data pointed out that E6/E7/LMP1 cooperation slightly deregulates the expression patterns of β-catenin and Erk1/Erk2, whereas it significantly induces the phosphorylation of both proteins in comparison with E6/E7 and LPM1 alone and with wild-type cells (Figure 7).

## Discussion

In this study, we investigated for the first time, the cooperative outcome of E6/E7 of HPV type 16 and LMP1 of EBV oncoproteins in two human breast cancer cell lines, MCF7 and MDA-MB-231, with regard to certain parameters related to cell proliferation, cell cycle progression, and colony formation, where HNME cells were used as control. Moreover, we explored the cooperative role of E6/E7 and LMP1 in cell motility and invasion as well as the expression patterns of EMT biomarkers, which are key regulators of cell invasion and metastasis (54). Our data showed clearly that E6/E7 of high-risk HPV type 16 can cooperate with LMP1 of EBV to enhance cell proliferation and deregulate cell cycle progression of MCF7, MDA-MB-231, and HNME cells; in addition, this cooperation stimulates colony formation of human breast cancer cells, but not in HNME cells, thus indicating its inability to provoke neoplastic transformation of human normal mammary cells.

The article "Oncoproteins of High-Risk HPV and EBV Cooperate to Enhance Cell Motility and Invasion of Human Breast Cancer Cells via Erk1/Erk2 and β-Catenin Signaling Pathways" was retracted in 2021. Reason: concerns about the images.

Several studies reported that high-risk HPVs can be presented in human breast cancer, especially types 16 and 18 that represent the most frequent HPV types worldwide (10, 14, 18, 32); in this context, it has been pointed out that HPV types 16 and 18 can promote breast carcinogenesis (55, 56). On the one hand, and similar to our present data, we have previously demonstrated that E6/E7 of HPV type 16 converts non-invasive and non-metastatic breast cancer cells into invasive and metastatic ones (38). On the other hand, numerous recent reports, including those from our laboratory, revealed that EBV can be detected in human breast cancer where it can play a vital role in the initiation and/or progression of this cancer (12, 14, 36). More recently, several investigations revealed that human oncoviruses, especially high-risk HPVs and EBV can be co-present in different types of human carcinomas, including cervical, head and neck, colorectal, and the breast (12, 14, 32, 36, 41–46). In this context, we have recently reported that high-risk HPVs and EBV are co-present in 32 and 47% of breast cancer samples from Syrian and Qatari women, respectively (14, 36); more significantly, our studies pointed out that the co-presence of these oncoviruses is associated with tumor grade and stage in addition to positive lymph nodes in examined breast cancer samples from Syria and Qatar (14, 36). However, the underlying molecular mechanisms behind high-risk HPVs and EBV oncoproteins interaction need to be identified. We herein explored the mechanism of HPV/EBV oncoproteins cooperation in breast cancer cell line models. It is worth noting that a previous study has shown a significant association between the co-presence of HPVs and EBV in luminal A and TNBC subtypes (36). Our present data revealed that the HPV/EBV cooperation enhances colony formation of luminal A and TNBC cancer cell lines, MCF7 and MDA-MB-231, respectively, which is a marker of cancer aggressiveness; it stimulates cell proliferation and deregulates cell cycle progression of these two breast cancer cell lines and HNME cells.

On other hand, it is well-known today that in cancer progression, EMT is a critical phenomenon characterized by the disruption of intracellular tight junctions as well as the loss of cell-cell contact (57). Moreover, in human carcinomas, cancer progression is accompanied by loss of E-cadherin and β-catenin in addition to enhanced expression of vimentin and fascin, thereby promoting EMT (57–60). In this investigation, we analyzed the effect of E6/E7 and LMP1 oncoproteins cooperation on the expression patterns of E-cadherin, β-catenin, vimentin, and fascin in luminal A and TNBC breast cancer cells (MCF7 and MDA-MB-231, respectively). We found that E6/E7/LMP1 downregulates the expression of E-cadherin and β-catenin, while vimentin and fascin are upregulated, thus indicating loss of cell–cell adhesion, especially E-cadherin/catenin complex. Our data are in concordance with previous studies, where the loss of E-cadherin expression is associated with EMT and promotes cells to develop an invasive phenotype (61, 62). While, an *in vivo* study in immune-deficient mice reported the loss of E-cadherin to promote tumorigenicity, EMT, and metastasis (63); another study by Kanai et al. (64) reported that loss of E-cadherin correlates with increased invasiveness and poorly differentiated breast carcinomas. On the other hand, in breast cancer, increased expression of vimentin and mesenchymal phenotypes correlates with more aggressive tumor characteristics (65). Thus, we herein show for the first time that E6/E7 of HPV type 16 cooperates with LMP1 of EBV to induce cell motility and invasion of the two human breast cancer cell lines, which is accompanied by the deregulation of EMT biomarkers. Regarding the molecular pathways of this cooperation, we assumed that β-catenin signaling pathways are involved in these events since β-catenin can act as a transcription regulator as well as a cell–cell adhesion molecule (66). Thus, it is plausible that the presence of these oncoproteins and their cooperation has an opposite effect on β-catenin pathways, particularly given their role in inducing β-catenin phosphorylation and inhibiting cell–cell adhesion leading to the enhancement of cell motility and invasion of MCF7 and MDA-MB-231 cell lines. Thus, our data indicate that the co-presence of these oncoviruses stimulates mesenchymal transition (EMT), thus promoting invasion and metastasis; concordantly, it is well-established that metastatic breast cancer is significantly associated with poor prognosis (67).

The article "Oncoproteins of High-Risk HPV and EBV Cooperate to Enhance Cell Motility and Invasion of Human Breast Cancer Cells via Erk1/Erk2 and β-Catenin Signaling Pathways" was retracted in 2021. Reason: concerns about the images.

Moreover, our data revealed that the E6/E7/LMP1 oncoproteins cooperation enhances the phosphorylation of β-catenin as well as Erk1/Erk2 pathway leading to loss of E-cadherin expression and causing a cascade of cellular process deregulations including proliferation, differentiation, motility, and invasion (68). Earlier studies showed that Erk1/Erk2 activation enhances cell motility and invasion of several types of human cancer cells, including breast (52–54, 69), which is in accordance with our present data. However, similar to our data, it has been shown that inactivation of Erk1/2 pathways can affect cell proliferation and cause G1 phase arrest (70, 71). Accordingly, in our cell line models, the ERK activity provoked by the E6/E7/LMP1 cooperation caused an increase in G0/G1 phase of the cell cycle.

## Conclusions

In conclusion, our data point out for the first time that oncoproteins of high-risk HPV and EBV cooperate to stimulate cell proliferation and deregulate cell cycle progression of human breast cancer and normal cells; more significantly, this crosstalk can enhance cell motility and invasion abilities of human breast cancer cells *via* β-catenin and Erk1/Erk2 signaling pathways. Nevertheless, future studies unraveling the mechanisms by which human oncoviruses, including HPV and EBV, endure and stimulate each other's virulence is a major step toward developing therapeutic strategies against human oncoviruses and their associated cancers.

## Data Availability Statement

The original contributions presented in the study are included in the article/supplementary material, further inquiries can be directed to the corresponding author/s.

## Author Contributions

A-EA and HA-T: conceptualization and resources. AJ and IG: methodology, validation, formal analysis, and data curation. AJ: software. IG: writing—original draft preparation. SV, A-EA, and HA-T: supervision, funding acquisition, and writing—review and editing. All authors have read and agreed to the published version of the manuscript.

## Conflict of Interest

The authors declare that the research was conducted in the absence of any commercial or financial relationships that could be construed as a potential conflict of interest.

## Abbreviations

DMEM: Dulbecco's modified Eagle's medium
DMSO: dimethyl sulfoxide
EBV: Epstein–Barr virus
ERK: extracellular signal-regulated kinases
FBS: fetal bovine serum
GAPDH: glyceraldehyde 3-phosphate dehydrogenase
HER2: human epidermal growth factor receptor-2
HNME: human normal mammary epithelial
HPV: human papillomavirus
LMP: latent membrane protein
MTT: 3-(4,5-dimethylthiazol-2-yl)-2,5-diphenyl tetrazolium bromide
ORF: open-reading frame
PBS: phosphate-buffered saline
Pen Strep: penicillin–streptomycin
RT-PCR: reverse transcription-polymerase chain reaction
TNBC: triple negative breast cancer.

## References

[1] FerlayJColombetMSoerjomataramIMathersCParkinDMPiñerosM. Estimating the global cancer incidence and mortality in 2018: GLOBOCAN sources and methods. Int J Cancer. (2019) 144:1941–53. 10.1002/ijc.3193730350310

[2] WeigeltBPeterseJLvan't VeerLJ. Breast cancer metastasis: markers and models. Nat Rev Cancer. (2005) 5:591–602. 10.1038/nrc167016056258

[3] Ala-EddinAl Moustafa AYGhabreauLMohamedAHAchkharA. Brain metastases progression of breast cancer. In: MehmetG, editor. Breast Cancer. London: Intech Open (2011).

The article "Oncoproteins of High-Risk HPV and EBV Cooperate to Enhance Cell Motility and Invasion of Human Breast Cancer Cells via Erk1/Erk2 and β-Catenin Signaling Pathways" was retracted in 2021. Reason: concerns about the images.

[4] Cancer Genome Atlas N. Comprehensive molecular portraits of human breast tumours. Nature. (2012) 490:61–70. 10.1038/nature1141223000897PMC3465532

[5] PerouCMSørlieTEisenMBvan de RijnMJeffreySSReesCA. Molecular portraits of human breast tumours. Nature. (2000) 406:747–52. 10.1038/3502109310963602

[6] ClausEBSchildkrautJMThompsonWDRischNJ. The genetic attributable risk of breast and ovarian cancer. Cancer. (1996) 77:2318–24. 10.1002/(sici)1097-0142(19960601)77:11<2318::Aid-cncr21>3.0.Co;2-z8635102

[7] CauchiJPCamilleriLScerriC. Environmental and lifestyle risk factors of breast cancer in Malta-a retrospective case-control study. EPMA J. (2016) 7:20. 10.1186/s13167-016-0069-z27679672PMC5029064

[8] LabrecqueLGBarnesDMFentimanISGriffinBE. Epstein-Barr virus in epithelial cell tumors: a breast cancer study. Cancer Res. (1995) 55:39–45. 7805038

[9] GlaserSLHsuJLGulleyML. Epstein-Barr virus and breast cancer: state of the evidence for viral carcinogenesis. Cancer Epidemiol. Biomarkers Prev. (2004) 13:688–97. 15159298

[10] AkilNYasmeenAKassabAGhabreauLDarnelADAl MoustafaAE. High-risk human papillomavirus infections in breast cancer in Syrian women and their association with Id-1 expression: a tissue microarray study. Br J Cancer. (2008) 99:404–7. 10.1038/sj.bjc.660450318648363PMC2527786

[11] GlennWKHengBDelpradoWIacopettaBWhitakerNJLawsonJS. Epstein-Barr virus, human papillomavirus and mouse mammary tumour virus as multiple viruses in breast cancer. PLoS ONE. (2012) 7:e48788. 10.1371/journal.pone.004878823183846PMC3501510

[12] AboulkassimTYasmeenAAkilNBatistGAl MoustafaA-E. Incidence of Epstein-Barr virus in Syrian women with breast cancer: a tissue microarray study. Hum Vaccin Immunother. (2015) 11:951–5. 10.1080/21645515.2015.100934225933186PMC4514243

[13] LawsonJSGlennWKSalyakinaDDelpradoWClayRAntonssonA. Human papilloma viruses and breast cancer. Front Oncol. (2015) 5:277. 10.3389/fonc.2015.0027726734565PMC4679879

[14] Al MoustafaA-EAl-AntaryNAboulkassimTAkilNBatistGYasmeenA. Co-prevalence of Epstein-Barr virus and high-risk human papillomaviruses in Syrian women with breast cancer. Hum Vaccin Immunother. (2016) 12:1936–9. 10.1080/21645515.2016.113925527082145PMC4964818

[15] LawsonJSGlennWK. Multiple oncogenic viruses are present in human breast tissues before development of virus associated breast cancer. Infect Agents Cancer. (2017) 12:55. 10.1186/s13027-017-0165-229075317PMC5644159

[16] de VilliersEMFauquetCBrokerTRBernardHUzur HausenH. Classification of papillomaviruses. Virology. (2004) 324:17–27. 10.1016/j.virol.2004.03.03315183049

The article "Oncoproteins of High-Risk HPV and EBV Cooperate to Enhance Cell Motility and Invasion of Human Breast Cancer Cells via Erk1/Erk2 and β-Catenin Signaling Pathways" was retracted in 2021. Reason: concerns about the images.

[17] KanCYIacopettaBJLawsonJSWhitakerNJ. Identification of human papillomavirus DNA gene sequences in human breast cancer. Br J Cancer. (2005) 93:946–8. 10.1038/sj.bjc.660277816222323PMC2361649

[18] AntonssonASpurrTPChenACFrancisGDMcMillanNASaundersNA. High prevalence of human papillomaviruses in fresh frozen breast cancer samples. J Med Virol. (2011) 83:2157–63. 10.1002/jmv.2222322012724

[19] XueSALampertIAHaldaneJSBridgerJEGriffinBE. Epstein-Barr virus gene expression in human breast cancer: protagonist or passenger? Br J Cancer. (2003) 89:113–9. 10.1038/sj.bjc.660102712838311PMC2394222

[20] FawzySSallamMAwadNM. Detection of Epstein-Barr virus in breast carcinoma in Egyptian women. Clin Biochem. (2008) 41:486–92. 10.1016/j.clinbiochem.2007.12.01718258188

[21] JoshiDQuadriMGanganeNJoshiRGanganeN. Association of Epstein Barr virus infection (EBV) with breast cancer in rural Indian women. PLoS ONE. (2009) 4:e8180. 10.1371/journal.pone.000818019997605PMC2782138

[22] LorenzettiMADe MatteoEGassHMartinezVazquez PLaraJGonzalezP. Characterization of Epstein Barr virus latency pattern in Argentine breast carcinoma. PLoS ONE. (2010) 5:e13603. 10.1371/journal.pone.001360321042577PMC2962632

[23] DeshpandeCGBadveSKidwaiNLongneckerR. Lack of expression of the Epstein-Barr virus (EBV) gene products, EBERs, EBNA1, LMP1, and LMP2A, in breast cancer cells. Lab Invest. (2002) 82:1193–9. 10.1097/01.lab.0000029150.90532.2412218080

[24] LindelKForsterAAltermattHJGreinerRGruberG. *Breast* cancer and human papillomavirus (HPV) infection: no evidence of a viral etiology in a group of Swiss women. Breast. (2007) 16:172–7. 10.1016/j.breast.2006.09.00117088061

[25] HachanaMZiadiSAmaraKToumiIKorbiSTrimecheM. No evidence of human papillomavirus DNA in breast carcinoma in Tunisian patients. Breast. (2010) 19:541–4. 10.1016/j.breast.2010.05.00720547456

[26] KadivarMMonabatiAJoulaeeAHosseiniN. Epstein-Barr virus and breast cancer: lack of evidence for an association in Iranian women. Pathol Oncol Res. (2011) 17:489–92. 10.1007/s12253-010-9325-z21207256

[27] YuYMorimotoTSasaMOkazakiKHaradaYFujiwaraT. Human papillomavirus type 33 DNA in breast cancer in Chinese. Breast Cancer. (2000) 7:33–6. 10.1007/BF0296718511029768

[28] Herrera-GoepfertRVela-ChávezTCarrillo-GarcíaALizano-SoberónMAmador-MolinaAOñate-OcañaLF. High-risk human papillomavirus (HPV) DNA sequences in metaplastic breast carcinomas of Mexican women. BMC Cancer. (2013) 13:445. 10.1186/1471-2407-13-44524083491PMC3852771

[29] IslamSDasguptaHRoychowdhuryABhattacharyaRMukherjeeNRoyA. Study of association and molecular analysis of human papillomavirus in breast cancer of Indian patients: Clinical and prognostic implication. PLoS ONE. (2017) 12:e0172760. 10.1371/journal.pone.017276028245287PMC5330495

The article "Oncoproteins of High-Risk HPV and EBV Cooperate to Enhance Cell Motility and Invasion of Human Breast Cancer Cells via Erk1/Erk2 and β-Catenin Signaling Pathways" was retracted in 2021. Reason: concerns about the images.

[30] SalmanNADaviesGMajidyFShakirFAkinrinadeHPerumalD. Association of high risk human papillomavirus and breast cancer: A UK based Study. Sci Rep. (2017) 7:43591. 10.1038/srep4359128240743PMC5378907

[31] KhodabandehlouNMostafaeiSEtemadiAGhasemiAPayandehMHadifarS. Human papilloma virus and breast cancer: the role of inflammation and viral expressed proteins. BMC Cancer. (2019) 19:61. 10.1186/s12885-019-5286-030642295PMC6332859

[32] GuptaIJabeenAAl-SarrafRFarghalyHVranicSSultaAA. The co-presence of high-risk human papillomaviruses and Epstein-Barr virus is linked with tumor grade and stage in Qatari women with breast cancer. Hum Vaccin Immunother. (2020) 17:1–8. 10.1080/21645515.2020.180297733006291PMC8018460

[33] KhanNACastilloAKoriyamaCKijimaYUmekitaYOhiY. Human papillomavirus detected in female breast carcinomas in Japan. Br J Cancer. (2008) 99:408–14. 10.1038/sj.bjc.660450218648364PMC2527789

[34] Al HamadMMatalkaIAl ZoubiMSArmogidaIKhasawnehRAl-HusainiM. Human mammary tumor virus, human papilloma virus, and Epstein-Barr virus infection are associated with sporadic breast cancer metastasis. Breast Cancer. (2020) 14:1178223420976388. 10.1177/117822342097638833281452PMC7691892

[35] YahiaZAAdamAAElgizouliMHusseinAMasriMAKamalM. Epstein Barr virus: a prime candidate of breast cancer aetiology in Sudanese patients. Infect Agents Cancer. (2014) 9:9–9. 10.1186/1750-9378-9-924607238PMC3975647

[36] GuptaINasrallahGKSharmaAJabeenASmattiMKAl-ThawadiHA. Co-prevalence of human Papillomaviruses (HPV) and Epstein-Barr virus (EBV) in healthy blood donors from diverse nationalities in Qatar. Cancer Cell Int. (2020) 20:107. 10.1186/s12935-020-01190-232265596PMC7118960

[37] NaushadWSurriyaOSadiaH. Prevalence of EBV, HPV and MMTV in Pakistani breast cancer patients: A possible etiological role of viruses in breast cancer. Infect Gene Evolut. (2017) 54:230–7. 10.1016/j.meegid.2017.07.01028705719

[38] YasmeenABismarTAKandouzMFoulkesWDDesprezP-YAl MoustafaA-E. E6/E7 of HPV type 16 promotes cell invasion and metastasis of human breast cancer cells. Cell Cycle. (2007) 6:2038–42. 10.4161/cc.6.16.455517721085

[39] HoriuchiKMishimaKIchijimaKSugimuraMIshidaTKiritaT. Epstein-Barr virus in the proliferative diseases of squamous epithelium in the oral cavity. Oral Surg Oral Med Oral Pathol Oral Radiol Endodontol. (1995) 79:57–63. 10.1016/S1079-2104(05)80075-77614163

[40] ShimakageMHoriiKTempakuAKakudoKShirasakaTSasagawaT. Association of Epstein-Barr virus with oral cancers. Hum Pathol. (2002) 33:608–14. 10.1053/hupa.2002.12978612152159

The article "Oncoproteins of High-Risk HPV and EBV Cooperate to Enhance Cell Motility and Invasion of Human Breast Cancer Cells via Erk1/Erk2 and β-Catenin Signaling Pathways" was retracted in 2021. Reason: concerns about the images.

[41] Al MoustafaA-EChenDGhabreauLAkilN. Association between human papillomavirus and Epstein-Barr virus infections in human oral carcinogenesis. Med Hypotheses. (2009) 73:184–6. 10.1016/j.mehy.2009.02.02519361933

[42] Al MoustafaAECyprianFSAl-AntaryNYasmeenA. High-risk human papillomaviruses and Epstein-Barr virus presence and crosstalk in human oral carcinogenesis. In: Al MoustafaAE, editor. Development of Oral Cancer: Risk Factors and Prevention Strategies. Cham: Springer International Publishing (2017). p. 83–94.

[43] Al-ThawadiHGhabreauLAboulkassimTYasmeenAVranicSBatistG. Co-incidence of Epstein-Barr virus and high-risk human papillomaviruses in cervical cancer of Syrian women. Front Oncol. (2018) 8:250. 10.3389/fonc.2018.0025030035100PMC6043788

[44] Al-ThawadiHGuptaIJabeenASkenderiFAboulkassimTYasmeenA. Co-presence of human papillomaviruses and Epstein–Barr virus is linked with advanced tumor stage: a tissue microarray study in head and neck cancer patients. Cancer Cell Int. (2020) 20:361. 10.1186/s12935-020-01348-y32774155PMC7397600

[45] GuptaIJabeenASkenderiFMalkiMIAl-ThawadiHAl MoustafaAE. High-risk human papillomaviruses (HPV) and Epstein - Barr virus (EBV) are commonly present in rectal cancer. Mod Pathol. (2020) 33:676. 10.3390/pathogens906045231673084

[46] MalkiMIGuptaIFernandesQAboulkassimTYasmeenAVranicS. Co-presence of Epstein-Barr virus and high-risk human papillomaviruses in Syrian colorectal cancer samples. Hum Vaccin Immunother. (2020) 16:2403–7. 10.1080/21645515.2020.172668032186955PMC7644212

[47] Al MoustafaAFoulkesWDBenlimameNWongAYenLBergeronJ. E6/E7 proteins of HPV type 16 and ErbB-2 cooperate to induce neoplastic transformation of primary normal oral epithelial cells. Oncogene. (2004) 23:350–8. 10.1038/sj.onc.120714814724563

[48] YasmeenAHoseinANYuQAl MoustafaA-E. Critical role for D-type cyclins in cellular transformation induced by E6/E7 of human papillomavirus type 16 and E6/E7/ErbB-2 cooperation. Cancer Sci. (2007) 98:973–7. 10.1111/j.1349-7006.2007.00504.x17489986PMC11158292

[49] YasmeenAAlachkarADekhilHGambacorti-PasseriniCAl MoustafaA-E. Locking Src/Abl tyrosine kinase activities regulate cell differentiation and invasion of human cervical cancer cells expressing E6/E7 oncoproteins of high-risk HPV. J Oncol. (2010) 2010:530130. 10.1155/2010/53013020862378PMC2938462

[50] YasmeenAZhangLAl MoustafaA-E. Does the vesicular stomatitis virus really have a selective oncolytic effect in human cancer? Int J Cancer. (2010) 126:2509–10. 10.1002/ijc.2492219795451

[51] GuptaIGhabreauLAl-ThawadiHYasmeenAVranicSAl MoustafaA-E. Co-incidence of human papillomaviruses and Epstein-Barr virus is associated with high to intermediate tumor grade in human head and neck cancer in Syria. Front Oncol. (2020) 10:1016. 10.3389/fonc.2020.0101632974123PMC7468388

The article "Oncoproteins of High-Risk HPV and EBV Cooperate to Enhance Cell Motility and Invasion of Human Breast Cancer Cells via Erk1/Erk2 and β-Catenin Signaling Pathways" was retracted in 2021. Reason: concerns about the images.

[52] CyprianFSAl-FarsiHFVranicSAkhtarSAl MoustafaA-E. Epstein-Barr virus and human papillomaviruses interactions and their roles in the initiation of epithelial-mesenchymal transition and cancer progression. Front Oncol. (2018) 8:111. 10.3389/fonc.2018.0011129765906PMC5938391

[53] SalehAIMohamedIMohamedAAAbdelkaderMYalcinHCAboulkassimT. Elaeagnus angustifolia plant extract inhibits angiogenesis and downgrades cell invasion of human oral cancer cells via Erk1/Erk2 Inactivation. Nutr Cancer. (2018) 70:297–305. 10.1080/01635581.2018.141247229300111

[54] Al MoustafaAEAchkharAYasmeenA. EGF-receptor signaling and epithelial-mesenchymal transition in human carcinomas. Front Biosci. (2012) 4:671–84. 10.2741/s29222202084

[55] PeranIRiegelADaiYSchlegelRLiuX. Is HPV-18 present in human breast cancer cell lines? Br J Cancer. (2010) 102:1549–52. 10.1038/sj.bjc.660567120407441PMC2869170

[56] WangYXLiYZZhangZYWangJQCuiJQianXL. HPV16 E6 promotes breast cancer proliferation via upregulation of COX-2 expression. Biomed Res Int. (2017) 2017:2948467. 10.1155/2017/294846729250535PMC5700552

[57] WuYSarkissyanMVadgamaJV. Epithelial-Mesenchymal transition and breast cancer. J Clin Med. (2016) 5:13. 10.3390/jcm5020013PMC477376926821054

[58] SatelliALiS. Vimentin in cancer and its potential as a molecular target for cancer therapy. Cell Mol Life Sci. (2011) 68:3033–46. 10.1007/s00018-011-0735-121637948PMC3162105

[59] MaoXDuanXJiangB. Fascin induces epithelial-mesenchymal transition of cholangiocarcinoma cells by regulating Wnt/β-catenin signaling. Med Sci Monit. (2016) 22:3479–85. 10.12659/msm.89725827680563PMC5045920

[60] XiaoCWuCHHuHZ. LncRNA UCA1 promotes epithelial-mesenchymal transition (EMT) of breast cancer cells via enhancing Wnt/beta-catenin signaling pathway. Eur Rev Med Pharmacol Sci. (2016) 20:2819–24. 27424981

[61] KimKLuZHayED. Direct evidence for a role of beta-catenin/LEF-1 signaling pathway in induction of EMT. Cell Biol Int. (2002) 26:463–76. 10.1006/cbir.2002.090112095232

[62] ThieryJP. Epithelial-mesenchymal transitions in tumour progression. Nat Rev Cancer. (2002) 2:442–54. 10.1038/nrc82212189386

[63] BirchmeierWBehrensJ. Cadherin expression in carcinomas: role in the formation of cell junctions and the prevention of invasiveness. Biochim Biophys Acta. (1994) 1198:11–26. 10.1016/0304-419x(94)90003-58199193

[64] KanaiYOdaTTsudaHOchiaiAHirohashiS. Point mutation of the E-cadherin gene in invasive lobular carcinoma of the breast. Jpn J Cancer Res. (1994) 85:1035–9. 10.1111/j.1349-7006.1994.tb02902.x7961105PMC5919349

[65] JørgensenCLTForsareCBendahlPOFalckAKFernöMLövgrenK. Expression of epithelial-mesenchymal transition-related markers and phenotypes during breast cancer progression. Breast Cancer Res Treat. (2020) 181:369–81. 10.1007/s10549-020-05627-032300922PMC7188722

The article "Oncoproteins of High-Risk HPV and EBV Cooperate to Enhance Cell Motility and Invasion of Human Breast Cancer Cells via Erk1/Erk2 and β-Catenin Signaling Pathways" was retracted in 2021. Reason: concerns about the images.

[66] HurJJeongS. Multitasking β-catenin: from adhesion and transcription to RNA regulation. Animal Cells Syst. (2013) 17:299–305. 10.1080/19768354.2013.853694

[67] WangRZhuYLiuXLiaoXHeJNiuL. The Clinicopathological features and survival outcomes of patients with different metastatic sites in stage IV breast cancer. BMC Cancer. (2019) 19:1091. 10.1186/s12885-019-6311-z31718602PMC6852913

[68] ToriiSYamamotoTTsuchiyaYNishidaE. ERK MAP kinase in G1 cell cycle progression and cancer. Cancer Sci. (2006) 97:697–702. 10.1111/j.1349-7006.2006.00244.x16800820PMC11158792

[69] Al MoustafaA-E. Epithelial-mesenchymal transition and its regulators are major targets of triple-negative breast cancer. Cell Adh Migr. (2013) 7:424–5. 10.4161/cam.2672824152786PMC3903687

[70] RooversKAssoianRK. Integrating the MAP kinase signal into the G1 phase cell cycle machinery. Bioessays. (2000) 22:818–26. 10.1002/1521-1878(200009)22:9<818::Aid-bies7>3.0.Co;2-610944584

[71] ZhengXOuYShuMWangYZhouYSuX. Cholera toxin, a typical protein kinase A activator, induces G1 phase growth arrest in human bladder transitional cell carcinoma cells via inhibiting the c-Raf/MEK/ERK signaling pathway. Mol Med Rep. (2014) 9:1773–9. 10.3892/mmr.2014.205424626525

